# Image Fusion Algorithm at Pixel Level Based on Edge Detection

**DOI:** 10.1155/2021/5760660

**Published:** 2021-08-09

**Authors:** Jiming Chen, Liping Chen, Mohammad Shabaz

**Affiliations:** ^1^School of Computer and Information Science, Hunan Institute of Technology, Hengyang 421002, China; ^2^Arba Minch University, Arba Minch, Ethiopia; ^3^Department of Computer Science Engineering, Chitkara University, Chandigarh, India

## Abstract

In the present scenario, image fusion is utilized at a large level for various applications. But, the techniques and algorithms are cumbersome and time-consuming. So, aiming at the problems of low efficiency, long running time, missing image detail information, and poor image fusion, the image fusion algorithm at pixel level based on edge detection is proposed. The improved ROEWA (Ratio of Exponentially Weighted Averages) operator is used to detect the edge of the image. The variable precision fitting algorithm and edge curvature change are used to extract the feature line of the image edge and edge angle point of the feature to improve the stability of image fusion. According to the information and characteristics of the high-frequency region and low-frequency region, different image fusion rules are set. To cope with the high-frequency area, the local energy weighted fusion approach based on edge information is utilized. The low-frequency region is processed by merging the region energy with the weighting factor, and the fusion results of the high findings demonstrate that the image fusion technique presented in this work increases the resolution by 1.23 and 1.01, respectively, when compared to the two standard approaches. When compared to the two standard approaches, the experimental results show that the proposed algorithm can effectively reduce the lack of image information. The sharpness and information entropy of the fused image are higher than the experimental comparison method, and the running time is shorter and has better robustness.

## 1. Introduction

Image fusion, as a visual data fusion technology, is one of the research focuses in the field of image fusion. It integrates many scientific and new technologies, such as sensor technology, image and signal processing, computer technology, artificial intelligence, statistics, and estimation theory [1–3]. Image fusion is to synthesize the image or image sequence information about a specific scene acquired by two or more sensors at the same time (or at different times) and to process the redundant or complementary multisource data in space or time according to certain rules to generate a new scene [4]. The explanation is more accurate and richer than any single data. The implementation of image fusion technology can overcome the limitations and differences in geometry, spectrum, and spatial resolution of images captured by a single sensor, enhance the reliability of images and the ability of image interpretation, and improve the ability of data classification and target recognition [5, 6].

Image fusion technology makes full use of redundant information and complementary information in a number of fused images. These characteristics make image fusion recognized in medicine, remote sensing, computer vision, meteorological forecast, military target monitoring, and recognition [7, 8]. On a variety of space and aviation carrier platforms, a variety of remote sensors are obtained. The fusion of a large number of remote sensing images with different spectra, bands, phases, and angles provides a good means for information fusion [9].

Relevant research at home and abroad is in the ascendant. Relevant research abroad originated in 1986. The U.S. Department of Defense and the U.S. Navy established the Data Fusion Subpanel (DFS). Since 1988, the United States has held an academic conference and published papers through SPIE. In 1977, the International Society of Information Fusion (ISIF) was established in the United States, and under the support by NASA (National Aeronautics and Space Administration) Ames Test Center, the U.S. Army Research Department, the IEEE Signal Processing Society, the IEEE Control Systems Society, and the IEEE Astronautical and Electronic Systems Society, an annual international information fusion conference was launched, so that scholars around the world can timely understand and grasp the new trends in the development of information fusion technology and promote the development of information fusion technology [10, 11]. Nowadays, scholars and technicians in the United States, Britain, Germany, France, Canada, Russia, Japan, India, and other countries are carrying out data fusion technology research.

Many scholars in China have done a lot of research on image fusion technology. In May 1995, the first special seminar on data fusion was held in Changsha, organized by the National Defense Science and Technology Commission. At present, some research institutes and high calibration institutes have actively carried out research work in this field, such as the Institute of Remote Sensing, Wuhan Surveying and Mapping Congress, Shanghai Institute of Technical Physics, Chinese Academy of Sciences, and Shanghai Jiaotong University [12]. From the current level of development, there is still a certain gap with the world level, there is less innovative work with unique ideas, mostly confined to the initial stage of theoretical research. The current image fusion algorithm at pixel level has low computational efficiency and large data storage and is affected by the accuracy of image registration, making that the image fusion at pixel level is poor in anti-interference and has limitations.

Fang et al. put forward an image fusion algorithm at pixel level based on spatial and spectral constraints [13]. Firstly, based on the hypothesis that the difference of each band before and after fusion is consistent with the observed spatial difference, the constraint term of spatial structure edge adaptation was proposed; then, based on the assumption that the relative relationship between the bands before and after fusion was invariant, the constraint term of the consistency of spectral band proportion was proposed; finally, the new constraint term was introduced into the variational model. The gradient descent method was used to solve the energy minimization problem, and the fusion result was obtained. The time-consuming process of image fusion was shorter, but the effect of image fusion was worse, the image definition was lower, and the image information loss was more. Gu et al. proposed a pixel-level image fusion algorithm based on block directional wavelet transform [14, 15]. The input image was evenly divided into several subblocks, and the directional wavelet of each image was determined by training; the sparse coefficients were obtained by the sparse transform of the image using the directional wavelet of the block, and the fusion coefficients were inversely transformed to obtain the fused image. The algorithm had a better image fusion effect, higher image clarity, and less information loss, but the running time was longer and the efficiency was lower. Zhao et al. proposed an image fusion algorithm of sparse representation at pixel level based on genetic algorithm optimization [16]. The fusion rules of sparse coefficients were determined by weighting coefficients, and the optimal weighting coefficients were solved by a genetic algorithm to realize the fusion of panchromatic and multispectral images at the pixel level. The image fusion effect of the algorithm was good, but the computation was large and the process was very complicated.

Based on the literature survey, it is found that there are various features of the images which may get altered during the fusion process of images. The distortion/alteration in the features of an image is not desirable. Hence, different kinds of algorithms are proposed by the various authors to overcome the above demerits. The current model is proposed with the objective to have better clarity, entropy, and lesser running time [17].

Through the study of relevant knowledge, aiming at the problems of current image fusion algorithm, an image fusion algorithm at pixel level based on edge detection is proposed. ROEWA algorithm is used for image edge detection, and variable precision fitting algorithm and edge curvature change are used to extract edge feature lines and angular points to enhance edge strength and improve image registration efficiency. Image fusion is realized by the energy fusion weighted method. Through simulation experiments, the proposed image fusion algorithm is compared with the method of literature, and the superiority of the proposed algorithm is verified.

## 2. Methods

Image fusion is not simple composition but emphasizes the optimization of information to highlight useful thematic information, eliminate or suppress irrelevant information, improve the image environment of target recognition, increase the reliability of interpretation, reduce ambiguity (i.e., ambiguity, incompleteness, uncertainty, and error), improve classification, and expand the scope of application and effect. The main purposes of image fusion are as follows:

1. Image sharpening
2. Improving the accuracy of geometric correction
3. Providing stereo observation capability for stereoscopic photography
4. Enhancing some of the characteristics of the data source of the original single sensor image
5. Improving the performance of detection, classification, understanding and recognition, and acquiring supplementary image data information
6. Using multitemporal data series to detect changes in scene and target
7. Using image information from other sensors to replace or compensate for image loss or fault information of a sensor
8. Overcoming the incompleteness of image data in object extraction and recognition

For the experimentation, the feature edge angle is the main parameter selected for investigation while the clarity, entropy, and running time are the main output parameter.

### 2.1. Image Edge Detection Based on ROEWA Operator

Edge detection is widely used in image segmentation, object recognition, and feature extraction. Before image registration and fusion, the ROEWA operator is used for image edge detection [18].

ROEWA operator is essentially an exponential smoothing filter based on linear minimum mean square error. The local mean of the detection window estimated by this filter is not an arithmetic mean, but an exponentially weighted mean. The expression of the filter is as given by

(1) $$\begin{array}{c} f\left(x\right)=K\;\exp\left(-a\left|x\right|\right), \end{array}$$

where *K* is the normalization constant and *a* is the filter coefficient. In discrete cases, *f*(*x*) can be implemented by filters *f*_1_(*x*) and *f*_2_(*x*), and the corresponding equation is as follows:

(2) $$\begin{array}{c} f\left(x\right)=\frac{1}{1+b}f_{1}\left(x\right)+\frac{b}{1+b}f_{2}\left(x-1\right), \end{array}$$

where *x*=1,2,…, *N*, and expressions of *f*_1_(*x*) and *f*_2_(*x*) are shown in equations (3) and (4), respectively,

(3) $$\begin{array}{c} f_{1}\left(x\right)=a\cdot b^{x}H\left(x\right), \end{array}$$

(4) $$\begin{array}{c} f_{2}\left(x\right)=a\cdot b^{-x}H\left(-x\right). \end{array}$$

In equations (3) and (4), 0 < *b* < 1, and *a*=1 − *b*; *H*(*x*) represents the Heaviside function. The expression of the function is given by

(5) $$\begin{array}{c} H\left(x\right)=\left\{\begin{array}{cc} 1, & x\geq 0,\\ 0, & x<0. \end{array}\right. \end{array}$$

For 2D image *I*(*x*, *y*), the edge strengths *R*_*X*_(*x*, *y*) and *R*_*Y*_(*x*, *y*) in the horizontal and vertical directions are calculated, respectively. In the horizontal direction, each column of the image is convoluted by a 1D smoothing filter *f*(*y*) and then convoluted by a filter *f*_1_(*x*) and a filter *f*_2_(*x*), respectively. The horizontal edge strengths *R*_*X*1_(*x*, *y*) and a filter *f*_2_(*x*) are obtained by a filter *f*_1_(*x*). The expression of the horizontal edge intensity *R*_*X*2_(*x*, *y*) of the image obtained is as follows:

(6) $$\begin{array}{c} R_{X1}\left(x,y\right)=f_{1}\left(y\right)*\left(f\left(x\right)⊙I\left(x,y\right)\right), \end{array}$$

(7) $$\begin{array}{c} R_{X2}\left(x,y\right)=f_{2}\left(y\right)*\left(f\left(x\right)⊙I\left(x,y\right)\right). \end{array}$$

In equations (6) and (7), *∗* and ⊙ are convolution symbols in the horizontal and vertical directions, respectively; for convolution results *s*_1_(*x*), *g*_2_(*x*), and *f*_2_(*x*) of given input signals *g*_1_(*x*) and *g*_2_(*x*) and *g*_1_(*x*) and *f*_1_(*x*), the corresponding equation is obtained by iteration. The corresponding equations are given by the following equations:

(8) $$\begin{array}{c} s_{1}\left(x\right)=g_{1}\left(x\right)*f_{1}\left(x\right)=a\left[g_{1}\left(x\right)-s_{1}\left(x-1\right)\right]+s_{1}\left(x-1\right),\;x=1,2,\ldots ,N, \end{array}$$

(9) $$\begin{array}{c} s_{2}\left(x\right)=g_{2}\left(x\right)*f_{2}\left(x\right)=a\left[g_{2}\left(x\right)-s_{2}\left(x-1\right)\right]+s_{2}\left(x-1\right),\;x=N,N-1,\ldots ,1. \end{array}$$

Convolution of *R*_*X*1_(*x*, *y*) and *R*_*X*2_(*x*, *y*) can also be calculated by using equations (8) and (9). By normalizing *R*_*X*1_(*x*, *y*) and *R*_*X*2_(*x*, *y*), the description of edge strength *R*_*X*_(*x*, *y*) in the horizontal direction of image *I*(*x*, *y*) can be obtained as represented in

(10) $$\begin{array}{c} R_{X}\left(x,y\right)=\max\left(\frac{R_{X1}\left(x,y\right)}{R_{X2}\left(x,y\right)},\frac{R_{X2}\left(x,y\right)}{R_{X1}\left(x,y\right)}\right). \end{array}$$

Similarly, the edge strength *R*_*Y*_(*x*, *y*) in the vertical direction of image *I*(*x*, *y*) can be obtained. According to *R*_*X*_(*x*, *y*) and *R*_*Y*_(*x*, *y*), the edge strength *r*(*x*, *y*) based on the ROEWA operator can be obtained as

(11) $$\begin{array}{c} r\left(x,y\right)=\sqrt{R_{X}^{2}\left(x,y\right)+R_{Y}^{2}\left(x,y\right)}. \end{array}$$

The calculation process of *r*(*x*, *y*) is further deduced, and the observational equations at pixel level [19] for the actual representation meanings and spatial coupling relationships of *R*_*X*1_(*x*, *y*), *R*_*X*2_(*x*, *y*), *R*_*Y*1_(*x*, *y*), and *R*_*Y*2_(*x*, *y*) components are obtained. Further derivation of equation (8), the derivation process of *s*_1_(*x*) is as shown in

(12) $$\begin{array}{c} s_{1}\left(x\right)=a\cdot g_{1}\left(x\right)+\left(1-a\right)\cdot s_{1}\left(x-1\right)\\ =a\cdot g_{1}\left(x\right)+\left(1-a\right)\cdot \left[a\cdot g_{1}\left(x-1\right)+\left(1-a\right)\cdot s_{1}\left(x-2\right)\right]\\ =\sum_{n=0}^{x-1}a{\left(1-a\right)}^{n}g_{1}\left(x-n\right). \end{array}$$

According to 1 − *a*=*b*, the expression of *s*_1_(*x*) can be obtained as follows :

(13) $$\begin{array}{c} s_{1}\left(x\right)=\sum_{n=0}^{x-1}ab^{n}g_{1}\left(x-n\right). \end{array}$$

Similarly, it can get the expression of *s*_2_(*x*) as shown as follows:

(14) $$\begin{array}{c} s_{2}\left(x\right)=\sum_{n=N-x}^{0}ab^{n}g_{2}\left(x+n\right). \end{array}$$

The horizontal edge of the image is divided into four regions, A1, A2, A3, and A4, and each region is weighted. The expressions of weighted edge strength *R*_*X*1_(*x*, *y*) and *R*_*X*2_(*x*, *y*) corresponding to the left and right regions in the horizontal direction are obtained as shown in

(15) $$\begin{array}{c} R_{X1}\left(x,y\right)=\frac{1}{1+b}\varphi_{1}\left(x,y\right)+\frac{b}{1+b}\varphi_{2}\left(x,y\right), \end{array}$$

(16) $$\begin{array}{c} R_{X2}\left(x,y\right)=\frac{1}{1+b}\varphi_{3}\left(x,y\right)+\frac{b}{1+b}\varphi_{4}\left(x,y\right), \end{array}$$

where *φ*_1_(*x*, *y*), *φ*_2_(*x*, *y*), *φ*_3_(*x*, *y*), and *φ*_4_(*x*, *y*) are the exponentially weighted mean corresponding to regions A1, A2, A3, and A4, respectively.

Similarly, the expressions of weighted edge strength *R*_*Y*1_(*x*, *y*) and *R*_*Y*2_(*x*, *y*) corresponding to the region on the upper and lower sides of the vertical direction are given by

(17) $$\begin{array}{c} R_{Y1}\left(x,y\right)=\frac{1}{1+b}\varphi_{1}\left(x,y\right)+\frac{b}{1+b}\varphi_{3}\left(x,y\right), \end{array}$$

(18) $$\begin{array}{c} R_{Y2}\left(x,y\right)=\frac{1}{1+b}\varphi_{2}\left(x,y\right)+\frac{b}{1+b}\varphi_{4}\left(x,y\right). \end{array}$$

According to the edge vector synthesis map of the ROEWA image and the normalization processing method, the vector sum |*r*_*x*_(*x*, *y*)| of *X*-axis direction and the vector sum |*r*_*y*_(*x*, *y*)| of *Y*-axis direction can be obtained as

(19) $$\begin{array}{c} \left|r_{x}\left(x,y\right)\right|=\left|r_{0}^{\prime }\right|-\left|r_{2}^{\prime }\right|, \end{array}$$

(20) $$\begin{array}{c} \left|r_{y}\left(x,y\right)\right|=\left|r_{1}^{\prime }\right|-\left|r_{3}^{\prime }\right|, \end{array}$$

where |*r*_0_′| and |*r*_2_′| are the normalized values of the positive and negative *X*-axis direction vectors, and |*r*_1_′| and |*r*_3_′| are the normalized values of the positive and negative *Y*-axis direction vectors, respectively.

The edge strength *r*_*e*_(*x*, *y*) of the image at the pixel level is obtained. The equation is given as follows:

(21) $$\begin{array}{c} r_{e}\left(x,y\right)=\sqrt{r_{x}^{2}\left(x,y\right)+r_{y}^{2}\left(x,y\right)}. \end{array}$$

The edge direction *D*_*e*_(*x*, *y*) of the image at the pixel level is obtained. The equation is given as follows:

(22) $$\begin{array}{c} D_{e}\left(x,y\right)=\langle r_{x}\left(x,y\right),r_{y}\left(x,y\right)\rangle \in \left[0,2\pi \right). \end{array}$$

Edge is the most basic feature of the image. It exists between target and background and between targets. If we can accurately extract the edge of the target and fuse different pattern images on this basis, the target in the fused image will be clear and easy to follow up processing.

### 2.2. Extraction of Feature Line and Angular Point of Image Edge

Edge provides a good feature for image registration, but it is difficult to translate into the mathematical language to make use of it. In order to facilitate the subsequent image fusion and improve the fusion efficiency, it is necessary to extract the feature lines and angular points of the image edge.

The characteristics of the edge lines are extracted. The edges are first fitted with variable precision lines, and then the edges are confidently evaluated. For picture registration, only the most valuable edge feature lines [20] are kept. The extraction process of specific features is as follows:

Supposing that the edge image is detected by edge detection, and the edge image *I*_*e*_ with a single-pixel width is obtained. If the pixel value of the edge point is 1 and the pixel value of the nonedge point is 0, then the specific process of fitting the edge image *I*_*e*_ is as follows:

1. Any edge *I*_*e*_^*i*^ in the image is extracted. If the relationship between edge length *L*_*e*_^*i*^ and the length of the line segment *L*_*s*_^*i*^ between the two endpoints satisfies *L*_*s*_^*i*^/*L*_*e*_^*i*^ ≥ *t*, 0 < *t* < 1, it is considered that the fitting is successful and the threshold *t* is the fitting precision
2. Otherwise, the most distant edge point is selected on the edge, and the original edge is divided into two edges together with the two edge endpoints. Repeat step 1 until the whole edge is completely fitted

The single edge can be obtained through the following three ways:

1. Isolated single edges: it can be obtained by tracking the edge endpoint to another endpoint; endpoint detection can be carried out by convoluting the image template with the edge map, and the edge point whose convolution result is “1” is an isolated single edge endpoint
2. Intersected edges: this kind of edge is formed by intersected several edges, and there are nodes, which can be obtained by tracking edge endpoints to nodes. Node detection examines the neighborhood of the current edge point clockwise. If the number of edges from the background to the edge is *n* ≥ 3, the edge point is the intersected edge node
3. Closed edges: it can select the two points with the largest distance between the edges and divide the closed edges into two edges.

According to the above steps, it can fit all the edges in the edge graph *I*_*e*_, and the length of the edge can be accurately calculated from the following:

(23) $$\begin{array}{c} L_{e}^{i}=\frac{\sum_{xy}\left(I_{e}^{i}*T\right)}{2}, \end{array}$$

where *T* represents the template image.

Influenced by noise, scale, rotation, and other factors, the original edge often breaks, so that the edge which could be fitted by a straight line can be divided into several straight lines. Therefore, the fitting conditions are satisfied:

1. The distance between ends is similar
2. The two straight lines with a smaller directional difference are connected to the same straight line

The new line's endpoints are chosen from the two ends of the two lines having the largest distance between them. The results of fitting straight lines at the different unclosed edge and closed edge thresholds are varied. The more the value, the more precise the fitting, but the greater the number of straight lines after fitting. The probability of the same edge appearing in different images is different when the scale and illumination condition of the fused image are different. If the edge appearing in one image does not appear in the other image, the edge will not only provide no useful information for registration but also easily cause dryness. This makes the importance of different edges and corresponding lines for fusion registration different. The longer the edge length is, the greater the contrast between the two gray levels is, the higher the probability of the edge and the corresponding line appearing repeatedly in different images is. For this reason, each line after edge fitting is given reliability to represent the confidence *R* of the fusion registration process on the line:

(24) $$\begin{array}{c} R=k_{1}\times \frac{L}{L_{\max}}+k_{2}\times \frac{c}{c_{\max}}, \end{array}$$

where 0 ≤ *R* ≤ 1, weight coefficients *k*_1_ and *k*_2_ satisfy *k*_1_+*k*_2_=1, *c* represents image edge contrast, *L* represents image edge line length, and *c*_max_ and *L*_max_ are the maximum of corresponding variables, respectively; that is, the maximum credibility is given to the whole image with the maximum contrast and line length. When the light changes, the edge contrast changes greatly relative to the length of the straight line, and the corresponding weight coefficient is *k*_1_ > *k*_2_.

According to the line reliability distribution map of the Lenna edge image, only a few lines have high reliability. Most of the low credibility lines are caused by noise, unstable edges, and edge turning [21]. If these low-confidence lines are used in the final image fusion and registration process, not only the computational efficiency is greatly reduced but also the really useful lines will be submerged. In order to improve the computational efficiency and fusion registration stability, the low-confidence lines are removed before the confidence assignment, and only the lines satisfying the following constraints are retained:

(25) $$\begin{array}{c} \left\{\begin{array}{c} l>\bar{l}+\sigma_{l},\\ c>\bar{c}+\sigma_{c}, \end{array}\right. \end{array}$$

where $\bar{l}$, *σ*_*l*_, $\bar{c}$, and *σ*_*c*_ represent the average value and standard deviation of line length and edge contrast, respectively.

According to the line set of the Lenna edge image, which is reserved and discarded after line fitting, it can be seen that the reserved line is clear and stable and can fully characterize the original image.

In order to further reduce the noise interference on the edge of the image, it is necessary to further adjust the edge. After adjusting, the basic structure of the image is represented by a few significant edges as possible. In image fusion, the repetitive detection rate of the same features in different images is very important to the stability of image fusion and registration. For edges, having a long length is the main feature of salient edges. This kind of edge has a high rate of repeated detection, while short edges are often caused by noise or unstable gray changes. According to the measurement results of each edge length in the edge image, only the edges whose length exceeds a certain threshold are retained.

The adjusted edge image can use a few significant edges to represent the basic structure of the image. In addition, at the angular point of the image edge and the intersection of multi-image edges, the edges no longer have the edge amplitude and direction, which makes the edges inevitably break and brings difficulties for the next edge angular point detection. In order to maintain the continuity of the edges, it is necessary to link the broken edges. The edge links can be realized simply by connecting two endpoints which are close to each other from the two edges.

An edge angular point is the edge point of an image whose curvature changes dramatically. Generally, the angular point is determined by calculating the gray gradient of the current point in multiple directions. Freeman chain code is used to describe the edge of the image, and the edge angular points [22] are obtained by curvature calculation of Freeman chain code.

The standard Freeman code takes 45 degrees as the boundary and encodes the edge into an integer sequence bit, namely, {*a*_*i*_, *i*=0,1,2,3,4,5,6,7}, according to the position relationship between the current edge point and the previous edge point on the same edge. However, the standard Freeman codes also have some shortcomings, mainly manifested in that the mutation of the coding sequence cannot always accord with the real edge curvature mutation. If the edges of the two fused images are {7070707070} and {7007007001}, respectively, the curvature of the edges of the corresponding standard Freeman codes will not change significantly, but the value of the standard Freeman codes will change greatly, so the improved Freeman codes are adopted. By a translation operation of improved Freeman, the code {*a*_1_*a*_2_ … *a*_*n*_} with a length of *n* is encoded and is recoded into sequence coordination {*b*_1_*b*_2_ … *b*_*n*_} using the following methods:

(26) $$\begin{array}{c} \left\{\begin{array}{c} b_{1}=a_{1},\\ b_{i}=q_{i}, \end{array}\right. \end{array}$$

where *q*_*i*_ is an integer, satisfying (*q*_*i*_ − *a*_*i*_)mod8=0, and making |*q*_*i*_ − *b*_*i*−1_| minimum, *i*=2,3,…, *n*. The improved edge codes are {7878787878} and {7887887889}, respectively. According to the corresponding graphics, the change of Freeman code value is more consistent with the actual curvature of the edge.

After obtaining the edge Freeman code, we directly use Freeman code to describe the edge angular point. Firstly, the curvature or curvature degree *Cr*(*i*) of the current edge point is expressed by the absolute value of the difference of the mean value by Freeman coding in a certain range on the edge curve where the current edge point is located.

(27) $$\begin{array}{c} Cr\left(i\right)=\left|\frac{1}{Lc}\overset{i-Lc}{\underset{j=i-1}{\sum }}b_{j}-\frac{1}{Lc}\overset{i-Lc}{\underset{j=i+1}{\sum }}b_{j}\right|, \end{array}$$

where *Lc* represents the detection scale, which is used to filter out tiny interference points on the edge. For the special case that the above-calculated values cannot reflect the degree of bending, the following equation is used to modify the results.

(28) $$\begin{array}{c} Cr\left(i\right)=\left\{\begin{array}{cc} Cr\left(i\right), & Cr\left(i\right)\leq 4,\\ 8-Cr\left(i\right), & Cr\left(i\right)>4. \end{array}\right. \end{array}$$

Through verification, the curvature obtained after modification is more in line with the actual situation. After modification, all points on each edge are traversed, and the edge points satisfying the following constraints are decided as feature angular points if and only if

1. The edge point curvature is larger than the given threshold
2. The curvature of the edge points is the local maximum at present

The first condition guarantees that the feature points are “characteristic” and the second condition guarantees that the feature points are “spaced.” According to the test results, the smaller the curvature threshold is, the more angular points detected are.

### 2.3. Image Fusion Algorithm at Pixel Level Based on Edge Detection

According to the degree of information abstraction, image fusion technology can be carried out by pixel level, feature level, and decision level in three different degrees. Fusion at pixel level directly fuses the collected data. Pixel points must be registered strictly to preserve more original image information and provide rich, accurate, and reliable information that other fusion layers cannot provide. It is conducive to further analysis and processing and understanding of the image and provides optimal decision-making and recognition performance. Commonly used methods are PCA (principal component analysis), IS (intensity-hue-saturation) transform, and multiresolution decomposition methods, such as pyramid algorithm and multiresolution wavelet transform [23].

Image fusion at the pixel level is the lowest level fusion, and it is also the basis of image fusion for feature-level and decision-level. Image fusion at pixel level has the largest amount of information and the most extensive application.

Fusion rules are a significant component in determining the ultimate fusion outcomes in image fusion algorithms at the pixel level, as well as the emphasis and complexity of this study topic. The wavelet transform's high-frequency coefficients play a crucial role in retaining the image's edge characteristics. Low-frequency coefficients determine the image's contour at the same time. The level of wavelet decomposition has a significant impact on the quality of the fused image. The more layers of the wavelet transform, the more details of fusion results will be rich, but not the more layers, the better. In fact, the decomposition and synthesis of wavelet transform are the division of frequency bands. The more layers of decomposition are, the more subbands are produced, and the higher frequency bands are divided. The signal output of the solution is used as the input of the next band decomposition, and the increase of the number of layers leads to the increase of the signal displacement; on the other hand, the wavelet decomposition and synthesis must carry on the boundary extension, the more layers lead to the greater boundary distortion, and the loss of information is the loss that the inverse wavelet transform cannot recover. The 3–5 tier is more appropriate [24].

In order to enhance the effect of image fusion and reduce the loss of image information, different fusion algorithms are used according to the different characteristics of the image in the high- and low-frequency domain. Firstly, the image is decomposed into three layers, the position of edge pixels in each layer is extracted, the edge images in two perpendicular directions of different decomposition layers and frequency domain images are obtained, and the feature lines and feature angular points of each decomposition layer are extracted. According to the difference of features, different methods are used to fuse, and then, the image details are combined. Finally, the fusion image is obtained by inverse wavelet transform.

Image contour and edge information mainly exist in the low-frequency part of the image, and this part of the image fusion is mainly based on the image contour and edge information as the main selection basis; image detail information mainly exists in the high-frequency part, and this part of the image fusion is mainly based on the image detail information as the main selection basis. The main process of image fusion is shown in Figure 1, which can get the contour and edge information of the image without losing the detail information. The process involves the first step as detection of low- and high-frequency regions of the images to be fused separately. Then, the fusion algorithm processes the high-frequency region of one image to that of another image, and similarly, the low-frequency region of one image is fused with the low frequency of other images. Then, finally, the high- and low-frequency regions of the fused image are combined into one image.

According to the edge features of images A and B, the high-frequency region of the image is determined, which is recorded as *F*_LH_*A*__ and *F*_LH_*B*__, respectively. The energy *E*_LH_ of the 5 *∗* 5 region centered on (*x*, *y*) is as given in

(29) $$\begin{array}{c} E_{\text{LH}}=\sum_{\left(x,y\right)\in N}F_{H_{I}}\left(x,y\right), \end{array}$$

where *F*_*H*_*I*__(*x*, *y*) represents the gray value of a pixel at a certain point in the high-frequency region. In the *M* × *N* area, the calculation equation of the regional spatial frequency *f*_LH_*I*__ of the horizontal high-frequency image is as given in

(30) $$\begin{array}{c} f_{{\text{LH}}_{I}}=\sqrt{{\text{RF}}_{{\text{LH}}_{I}}^{2}+{\text{CF}}_{{\text{LH}}_{I}}^{2}}, \end{array}$$

where RF_LH_*I*__ is the row frequency and CF_LH_*I*__ is the column frequency.

When *a* = 1, the calculation process of the fusion horizontal high-frequency component *f* is as follows:

(1) If point (*x*, *y*) is completely at the edge of the horizontal high-frequency image, then it is given by
  (31) $$\begin{array}{c} F_{\text{CLH}}\left(x,y\right)=F_{{\text{LH}}_{A}}\left(x,y\right). \end{array}$$
(2) If point (*x*, *y*) is near the edge point of the horizontal high-frequency image, then it is represented by
  (32) $$\begin{array}{c} F_{\text{CLH}}\left(x,y\right)=\left\{\begin{array}{c} F_{{\text{LH}}_{A}}\left(x,y\right),\;f_{{\text{LH}}_{A}}\left(x,y\right)\geq \alpha f_{{\text{LH}}_{B}}\left(x,y\right),\\ \beta F_{{\text{LH}}_{A}}\left(x,y\right)+\alpha F_{{\text{LH}}_{B}}\left(x,y\right),\;f_{{\text{LH}}_{A}}\left(x,y\right)<f_{{\text{LH}}_{B}}\left(x,y\right). \end{array}\right. \end{array}$$
(3) If point (*x*, *y*) is away from the edge point of the horizontal high-frequency image, then then it is represented by

(33) $$\begin{array}{c} F_{\text{CLH}}\left(x,y\right)=\left\{\begin{array}{c} \alpha F_{{\text{LH}}_{A}}\left(x,y\right)+\beta F_{{\text{LH}}_{B}}\left(x,y\right),\;f_{{\text{LH}}_{A}}\left(x,y\right)\geq f_{{\text{LH}}_{B}}\left(x,y\right),\\ \beta F_{{\text{LH}}_{A}}\left(x,y\right)+\alpha F_{{\text{LH}}_{B}}\left(x,y\right),\;f_{{\text{LH}}_{A}}\left(x,y\right)<f_{{\text{LH}}_{B}}\left(x,y\right). \end{array}\right. \end{array}$$

In equations (32) and (33), *α* and *β* are weighting coefficients, satisfying 0 < *β* < *α* < 1 and *β*+*α*=1. Similarly, *F*_CLH_(*x*, *y*) and other high-frequency components at *E*_LH_*A*__ < *E*_LH_*B*__ can be obtained, and the obtained component results are fused to obtain a fusion result of the high-frequency region of the image, and the detailed information can be retained while the redundant detail information can be suppressed.

According to the characteristics of the low-frequency regions of the obtained images A and B, the low-frequency regions of the image are determined, denoted as *F*_LL_*A*__ and *F*_LL_*B*__, and the low-frequency region fusion process is as follows:

(1) Using the regional energy algorithm, the initial fusion of the low-frequency regions of images A and B is performed. The energy *E*_LL_ of the 5 × 5 region centered on (*x*, *y*) is calculated as given in
  (34) $$\begin{array}{c} E_{\text{LL}}=\sum_{\left(x,y\right)\in N}F_{L_{I}}\left(x,y\right), \end{array}$$
where *F*_*L*_*I*__(*x*, *y*) is the gray value of a pixel in the low-frequency region. The expression of the fused low-frequency component *F*_CL1_(*x*, *y*) is as given in
  (35) $$\begin{array}{c} F_{\text{CL}1}\left(x,y\right)=\left\{\begin{array}{cc} F_{L_{A}}\left(x,y\right), & E_{{\text{LL}}_{A}}\geq E_{{\text{LL}}_{B}},\\ F_{L_{B}}\left(x,y\right), & E_{{\text{LL}}_{A}}<E_{{\text{LL}}_{B}}. \end{array}\right. \end{array}$$
With the above method, the contour information and edge features of the image are better preserved.
(2) Using the weighting factor algorithm, the low-frequency regions of images A and B are fused again, and the low-frequency components are adjusted and fused by equation (36) to ensure the quality of the restored images is represented by
  (36) $$\begin{array}{c} F_{\text{CL}2}=\alpha \left|F_{L_{A}}\left(x,y\right)+kF_{L_{B}}\left(x,y\right)\right|-\beta \left|F_{L_{A}}\left(x,y\right)-kF_{L_{B}}\left(x,y\right)\right|. \end{array}$$
In the above equation, *k*, *α*, and *β* are weighting factors. *α*|*F*_*L*_*A*__(*x*, *y*)+*kF*_*L*_*B*__(*x*, *y*)| denotes the weighted mean of the images A and B, which affects the energy of the merged image, and plays a decisive role in the brightness of the merged image. *β*|*F*_*L*_*A*__(*x*, *y*) − *kF*_*L*_*B*__(*x*, *y*)| represents the weighted difference between images A and B, including the fuzzy information of the image. The factor *k* is mainly used to adjust the dominant ratio of images A and B so that the images with different brightness are balanced. The brightness of the image increases as the factor *α* increases, and the edge intensity of the image increases as the factor *β* increases [25]. For different images, the factor values can be adjusted appropriately to eliminate the blurred edges, ensuring that the edge information is not excessively lost during the subtraction.
(3) The pixel values of the fused images obtained by the two algorithms are compared, and the largest pixel value (or coefficient) is selected as the pixel value of the final fused image. The fusion rules are represented by

(37) $$\begin{array}{c} F_{\text{CL}}\left(x,y\right)=\left\{\begin{array}{cc} F_{\text{CL}1}\left(x,y\right), & F_{\text{CL}1}\left(x,y\right)\geq F_{\text{CL}2}\left(x,y\right),\\ F_{\text{CL}2}\left(x,y\right), & F_{\text{CL}1}\left(x,y\right)<F_{\text{CL}2}\left(x,y\right). \end{array}\right. \end{array}$$

Here, *F*_CL_(*x*, *y*) is the approximation coefficient of the fused image in the low-frequency region of the image.

According to the approximate coefficients of the low-frequency region and the fusion coefficient of the high-frequency regions, the fused image of each region is obtained by inverse wavelet transform, and the fused image of the obtained high-frequency region and low-frequency region is reconstructed to obtain a global fused image containing comprehensive information [26].

## 3. Results

In order to prove the validity and feasibility of the image fusion algorithm at pixel level based on edge detection, a simulation experiment is carried out. In the experiment, the clarity, entropy, and running time of the fused image are compared. The simulation experiment environment is as follows: MATLAB R2011a software, Intel Pentium Dual-Core E5300 processor, basic frequency at 2.60 GHz, 4 GB memory, Windows XP SP3 system. And the simulation data set My-Sea is selected as the basic data set, and the data is analyzed by the online data analysis software MOA (an experimental tool for massive online analysis).

The proposed image fusion algorithm at pixel level based on edge detection, the algorithm based on space and spectral constraints, and the algorithm based on block directional wavelet transform are used in this experiment. The experimental results are shown in the tables and figures. FA1 represents the image fusion algorithm based on edge detection, FA2 represents the algorithm based on spatial and spectral constraints, and FA3 represents the algorithm based on block directional wavelet transform.

Three kinds of image fusion algorithms are used to experiment, and a group of images are randomly selected as experimental samples [27, 28]. Three image fusion algorithms are used to extract five edge feature angular points, and the relative distance between the obtained edge angular points and the fitted line is calculated. The experimental results are shown in Figure 2. The abscissa of Figure 2 is the number of the extracted edge feature angular points, and the ordinate is the relative distance in units of *μ*m. The figure shows that the relative distance varies with the number of extracted edge feature angular points. It is noticed that the fusion algorithm FA2 has the highest value of relative distance as 7.55 *μ*m and FA1 has the least values of relative distance as 0.18 *μ*m for edge angle values of 3 and 4, respectively.

Through the image fusion and information entropy, the fusion performance of different image fusion algorithms is quantitatively evaluated. In the experiment, two sets of image sequences are randomly selected as experimental samples [29]. In order to improve the reliability of the experimental results, five experiments are performed using three image fusion algorithms, and the average of the sharpness and information entropy of each fusion image is taken as the experimental result. The sharpness and information entropy of the fused image obtained by each algorithm are shown in Tables 1 and 2.

According to the running time of the image fusion process of the three algorithms, the fusion efficiency of each image fusion algorithm is evaluated. In the experiment, the image samples in the performance comparison experiment are still selected for the experiment, and the running time of each image fusion algorithm is compared. The experimental results are shown in Table 3. The running time in Table 3 is the average of experimental results in 5 times.

## 4. Discussion

According to Figure 2, for the single feature angular point, the distance between the edge angular point 1 and the fitting lines is 1.15 *μ*m, 5.11 *μ*m, and 3.67 *μ*m, extracted by the proposed image fusion algorithm, the algorithm based on spatial and spectral constrained, and the algorithm based on block directional wavelet transform, respectively. The error of the proposed algorithm is the smallest. Compared with other feature angular points, the conclusion can be verified [30]. Combining the edge points of all image edges, the distance between the edge angle and the fitted line extracted by the proposed image fusion algorithm, the algorithm based on the spatial and spectral constraint, and the algorithm based on block directional wavelet transform is 0.18–1.51 *μ*m, 2.95–7.55 *μ*m, and 3.31–5.11 *μ*m, respectively [31, 32]. According to the above data, the edge detection and fitting effect of the proposed algorithm are better, and the location accuracy of edge feature angular is higher.

Analyzing the data in Tables 1 and 2, it can be seen that for sample group 1, compared with the image fusion algorithm at pixel level based on spatial and spectral constraints and algorithm based on block directional wavelet transform [33, 34], the obtained resolution is improved by 1.23 and 1.01 by using the proposed image fusion algorithm, and the information entropy content is higher by 0.82 and 0.47. According to the above data, the proposed algorithm has a better image fusion effect and higher image clarity and information content.

Analyzing the data in Table 3, for sample group 1, the running time of the proposed image fusion algorithm is 1.24 s less than the algorithm based on spatial and spectral constraints, and 3.11 s less than the algorithm based on block directional wavelet transform. According to the above data analysis results, the proposed algorithm takes the shortest time, which indicates that the proposed algorithm has higher fusion efficiency.

## 5. Conclusions

Image edge detection and image fusion are two important and closely related research directions in the field of image processing. They are of great significance for visual detection, target recognition, and image synthesis. The edge is the most significant part of the image local intensity change, with high stability, and is a prominent feature of the image. Image fusion is mainly used for practical problems such as multisource data fusion, time-series image analysis, target change detection, target recognition, and image mosaic.

In order to solve the problems of low efficiency, long running time, loss of image details, and poor fusion effect of traditional image fusion methods, a pixel-level image fusion algorithm based on edge detection is proposed. The achieved results are as follows:

1. Through the in-depth study and analysis of the ROEWA algorithm, the convolution process of the algorithm is further deduced, and the observation equation of each component of the image at the pixel level is obtained. Also, the image edge is weighted by region division to improve the image edge intensity.
2. According to the fitting calculation result and the curvature change of the edge angular point, the edge feature line and the feature angular point of the image are extracted, and the fitting threshold is adjusted appropriately to enhance the precision of the image registration and the fitting effect.
3. The wavelet transform algorithm is adopted, the fusion rules of the high-frequency region and the low-frequency region of the image are, respectively, set, and the regional energy algorithm is used for fusion to ensure the image fusion effect and avoid the loss of image detail information.
4. Fusion algorithm FA2 has the highest value of relative distance as 7.55 *μ*m and FA1 has the least values of relative distance as 0.18 *μ*m for edge angle values of 3 and 4, respectively.
5. Based on Tables 1–3, it is concluded that the fusion algorithm FA1 has the best sharpness of 5.18 and best entropy of 6.95 with the least run time of 5.98 seconds.

Although the performance of the image fusion algorithm has improved, there are still deficiencies. In the future stage, the imaging principle of various images will be deeply studied, the image features will be further subdivided, the edge positioning accuracy will be improved, and the edge detection efficiency will be improved. The real-time image fusion algorithm will be studied, and the parallel structure of image processing will be introduced into the image fusion algorithm, to enhance the real-time performance of image fusion.

## Figures and Tables

**Figure 1:** Flow chart of image fusion algorithm.

**Figure 2:** The extracted distance between the edge feature angular point and the fitted line by each image fusion algorithm.

**Table 1:** Comparison of the sharpness of the fused images by each image fusion algorithm.

Samples	Image fusion algorithm	Sharpness
Group 1	FA3	3.86
	FA2	3.64
	FA1	4.87

Group 2	FA3	4.11
	FA2	4.01
	FA1	5.18

**Table 2:** Comparison of information entropy of fused images by image fusion algorithms.

Samples	Image fusion algorithm	Information entropy
Group 1	FA3	6.36
	FA2	6.01
	FA1	6.83

Group 2	FA3	6.52
	FA2	6.43
	FA1	6.95

**Table 3:** Comparison of running time by each image fusion algorithm.

Samples	Image fusion algorithm	Running time (s)
Group 1	FA3	8.14
	FA2	6.27
	FA1	5.03

Group 2	FA3	9.06
	FA2	7.55
	FA1	5.98

## Data Availability

Data will be made available on request to the corresponding author.
